# The Low Endometrial Expression of Long Non-Coding RNA NORAD Is Associated with Recurrent Pregnancy Losses and Unexplained Infertility

This article has been retracted.

**DOI:** 10.1155/2022/6448666

**Published:** 2022-10-13

**Authors:** Ying Huang, Chengyong Wu, Chunmei Wei, Yekun Chen, Fei Xing

**Affiliations:** ^1^Department of Reproductive Medicine, Yichun People's Hospital, Yichun, Jiangxi 336000, China; ^2^Department of Clinical Laboratory, Huai'an Second People's Hospital and The Affiliated Huai'an Hospital of Xuzhou Medical University, Huai'an, Jiangsu 223001, China

## Abstract

**Objective:**

Unexplained infertility (UIF) or recurrent pregnancy loss (RPL) affects 10%–15% of couples in their reproductive years and is multifactorial and not completely elucidated. In this study, we attempt to determine the endometrial expression pattern of non-coding RNA activated by DNA damage (NORAD) in women with UIF and RPL, as well as its clinical significance.

**Methods:**

The microarray dataset GSE165004 was used to identify differentially expressed RNAs in the endometrial samples between women with RPL and fertile women and between women with UIF and fertile women. A total of 142 women were included in this retrospective analysis, including 32 women with UIF, 48 women with RPL, and 62 fertile women. The relative expression level of NORAD in the endometrial tissues was quantified by qRT-PCR.

**Results:**

NORAD stood out as an only overlapped lncRNA among differentially expressed RNAs in the endometrial samples between RPL and fertile women and between UIF and fertile women. It was showed that the endometrial tissues of UIF and RPL both were demonstrated with lower relative expression levels of NORAD (UIF: 2.09 ± 0.68; RPL: 1.98 ± 0.65) than the endometrial tissues of normal fertility (4.32 ± 1.04) (*P* < 0.001). Pearson correlation analysis demonstrated that the serum level of E2 was negatively correlated with the relative expression level of NORAD in the endometrial tissues of UIF (*r* = −0.630) and RPL (*r* = −0.696). Results of ROC curves showed that the endometrial expression of NORAD could be used to differentiate RPL and UIF with an AUC of 0.977 (95% CI: 0.956–0.999) and 0.970 (95% CI: 0.941–0.998), sensitivity of 0.873 and 0.955, and specificity of 0.845 and 0.948, respectively.

**Conclusion:**

The findings obtained from the study showed that the low endometrial expression of NORAD was linked to fertility-related problems, such as UIF and RPL.

## 1. Introduction

Infertility refers to the inability to establish clinical pregnancy after 1 year of regular and unprotected sexual intercourse, affecting 10–15% of reproductive-aged couples worldwide [1]. Approximately 72.4 million populations are estimated to suffer from infertility and 40.5 million people are currently seeking medical care [2]. Identifiable causes, such as ovulatory dysfunction, male factor infertility, and tubal disease, have been confirmed in 85% of those who experience infertility. Unexplained infertility (UIF) exists in the remaining 15% of infertile couples [3]. No direct explanations are identified in the couples with UIF presenting normal spermatogenesis and ovulation. Despite extensive research on unexplained infertility has been explored for decades, UIF still remains to a great extent unexplained [4]. Recurrent pregnancy loss (RPL) is a painful pregnancy disorder. It is defined as a failure of spontaneous pregnancy clinically recognized twice or more before 20–24 weeks of gestation including embryo and fetal loss but excludes ectopic pregnancies and molar pregnancies [5]. The progress in predicting and preventing RPL has been advanced. However, the diagnosis of RPL remains difficult due to its highly variable clinical manifestations and the uncertainty of pathogenesis [6].

Infertility in female is extremely heterogeneous in etiology, which may be due to complex interaction female development, hormone, and environment and genetic factors [7]. The non-coding RNA does not have the ability to encode proteins but contains information and function. These RNAs regulate gene expression in physiology and development including chromatin structure or epigenetic memory and transcription through activating or inactivating internal signals [8]. Non-coding RNA activated by DNA damage (NORAD) also known as LINC00657 is a highly conserved long non-coding RNA (lncRNA) compared to other lncRNAs, which is profusely expressed in a great quantity of cells due to DNA damage. Considerable studies revealed that NORAD has been involved in numerous processes concerning cancer promotion, such as cell proliferation, apoptosis, invasion, and metastasis. It may be a potential biomarker in pancreatic cancer, lung cancer, and colorectal cancer by regulating the downstream mechanisms [8, 9]. Another study demonstrated that lower expression of NORAD was detected in the breast milk exosomes of mothers of preterm infants compared with mothers who gave birth at term. It suggested that NORAD participated in the early human development [10]. The functional role of NORAD in female infertility is unclear at present. Therefore, this study recruited females with RPL or UIF and fertile females to explore the impacts of NORAD on occurrence of RPL or UIF and provide some evidences for clinical treatment.

## 2. Materials and Methods

### 2.1. GEO2R Bioinformatics Analysis

A microarray dataset deposited in the Gene Expression Omnibus (https://www.ncbi.nlm.nih.gov/gds, submission date: Jan 2021) and accessioned as GSE165004 was used to identify differentially expressed RNAs. This dataset was generated on the GPL16699 platform and contained endometrial samples from 24 women with RPL, 24 women with UIF, and 24 fertile women at days 19–21 of the menstrual cycle. Differentially expressed RNAs in the endometrial samples between women with RPL and fertile women and between women with UIF and fertile women were, respectively, sorted using the online tool GEO2R [11] based on the R software limma package. Sorted differentially expressed RNAs must fulfill log2|fold change (FC)| > 1 and adjusted *P* < 0.05.

### 2.2. Study Subjects

This retrospective study included women diagnosed with either UIF or RPL with no offspring from spontaneous pregnancies in our infertility center between January 2020 and December 2021. Women were diagnosed with UIF after routine fertility tests showing (i) infertility of more than 12 months, (ii) normospermic male partner according to the World Health Organization (2010) criteria [12], (iii) regular menstrual cycle of 25–35 days, positive ovulation tests, and/or progesterone levels ≥ 25 mmol/l, (iv) normal uterine cavity and bilateral tubal patency on the hysterosalpingogram or laparoscopy, and (v) normal hormonal tests (follicle stimulating hormone (FSH) ≤ 13 UI/l and anti-Müllerian hormone (AMH) ≥ 0.4 ng/ml) [13]. Women were diagnosed with RPL if they failed to conceive after ≥2 fresh IVF-ET/ICSI (in vitro fertilization-embryo transfer cycles/intracytoplasmic sperm injection) or had ≥3 consecutive miscarriages occurring before 20 weeks of gestation, documented by ultrasonography or histopathological examination. Eligible women with either UIF or RPL must have age between 18 and 40 years and detailed reports of laparoscopy and hysteroscopy (done within 1 month) and sign a written consent to participate in the study. Those with an identifiable cause of reproductive failure such as chromosomal abnormalities or anatomic defects identified on initial screen, with known endometriosis, adenomyosis, endocrine disorders (polycystic ovary syndrome), autoimmune diseases, or thrombophilia (inherited or acquired), with previous use of hormone therapy, with severe obesity (body mass index (BMI) > 35), or using antibiotics within at least two weeks before sample collection were excluded from this retrospective analysis. Women undergoing dilatation and curettage in our hospital at the same period, with regularly cycling women, at least one live birth, no history of infertility/treatment, no previous miscarriages and no associated gynecologic (endometriosis, fibroids, active or history of pelvic inflammatory disease) or other medical comorbidities such as hyperprolactinemia and thyroid disease were served as fertile controls. The study was approved by the Ethics Committee of our hospital.

### 2.3. Endometrial Sample Collection

Endometrial tissue was obtained from included women in 7–9 days after the luteinizing hormone surge detected using urine luteinizing hormone tests at the time of their medically indicated hysteroscopic endometrial biopsy or endometrial curettage.

### 2.4. RNA Extraction and Quantitative Real-Time PCR (qRT-PCR)

Total RNA was extracted from obtained endometrial tissues using the TRIzol reagent (Invitrogen, Carlsbad, CA, USA) following the manufacturer's manual. The generation of complementary DNA (cDNA) template was carried out using the PrimeScript RT Reagent kit (Takara, Dalian, China) following the manufacturer's manual. The qPCR was carried out using the SYBR® Premix Ex Taq™ II kit (Takara) and a ABI PRISM®7500 System (Applied Biosystems, Foster City, CA, USA) under the thermocycling conditions (95°C for 5 min, followed by 40 cycles at 95°C for 15 s, 60°C for 30 s, and 72°C for 1 min). The primer sequence information of NORAD was 5′-AAGCTGCTCTCAACTCCACC-3' (forward) and 5′-GGACGTATCGCTTCCAGAGG-3' (reverse), and that of GAPDH was 5′-GGAGCGAGATCCCTCCAAAAT-3' (forward) and 5′-GGCTGTTGTCATACTTCTCATGG-3' (reverse). The cycle threshold (Ct) values were normalized to the level of GAPDH, and results were then converted into fold change using the 2^−ΔΔCt^ formula.

### 2.5. Enzyme-Linked Immunosorbent Assay (ELISA)

All included women were subjected to venous blood collection in the morning for detection of serum levels of hormones including FSH, estradiol (E2), progesterone (P), luteinizing hormone (LH), testosterone (T), and prolactin (PRL) by ELISA methods. All ELISA procedures were performed in accordance with the protocol supplied by the kits' manufactures (R&D Systems, USA).

### 2.6. Statistical Analysis

Statistical analysis and figure creation were performed using GraphPad Prism 8 (GraphPad Software, CA, USA) and SPSS version 22.0 statistical package (IBM Corp, Armonk, NY, USA). Categorical data were shown by number with percentage and analyzed by chi-square test or Fisher's exact test (*P* < 0.05 regarded as significant difference). Measurement variables normally distributed are shown as mean ± standard deviation and analyzed by independent Student's *t*-test (*P* < 0.05 regarded as significant difference). The Pearson correlation test was used to assess the association between NORAD and serum levels of E2 and P. The receiver operating characteristic (ROC) and logistic regression analysis were performed to estimate the diagnostic values of NORAD in UIF and RPL.

## 3. Results

### 3.1. NORAD as a Differentially Expressed lncRNA in RPL and UIF

After GEO2R bioinformatics analysis, we identified six downregulated RNAs (log2FC > 1 and *P* < 0.05) in the endometrial samples between women with RPL and fertile women and three differentially expressed RNAs (two downregulated RNAs and an upregulated RNA, log2|FC| > 1 and *P* < 0.05) in the endometrial samples between women with UIF and fertile women (Table 1). NORAD stood out as an only overlapped lncRNA among differentially expressed RNAs in the endometrial samples between RPL and fertile women and between UIF and fertile women.

### 3.2. Demographics and Clinical Characteristics of Included Women

A total of 142 women were included in this retrospective analysis, including 32 women with UIF, 48 women with RPL, and 62 fertile women. Demographics and clinical characteristics of three groups of women are listed in Table 2, showing no significant difference on age, body mass index (BMI), the proportions of history of taking oral contraceptives, algomenorrhea, and family history among them. Of note, the serum levels of FSH, LH, T, PRL, and E2 were higher but the serum level of P was lower in women with either UIF or RPL than those in fertile women (*P* < 0.05). No significant difference was noted in these serum levels of hormones between the women with UIF and those with RPL (*P* > 0.05).

### 3.3. Low Endometrial Expression of NORAD in RPL and UIF

The relative expression level of NORAD in the endometrial tissues obtained from 32 women with UIF, 48 women with RPL, and 62 fertile women was quantified by qRT-PCR. It was showed that the endometrial tissues of UIF and RPL both were demonstrated with lower relative expression levels of NORAD (UIF: 2.09 ± 0.68; RPL: 1.98 ± 0.65) than the endometrial tissues of normal fertility (4.32 ± 1.04) (*P* < 0.001, Figure 1(a)). No evident significance was noted in the endometrial expression of NORAD between UIF and RPL (*P* > 0.05). Pearson correlation analysis demonstrated that the serum level of E2 was negatively correlated with the relative expression level of NORAD in the endometrial tissues of UIF (Figure 1(b), *r* = −0.630) and RPL (Figure 1(c), *r* = −0.696), but the serum levels of FSH, LH, T, PRL, and P were not correlated (*P* > 0.05).

### 3.4. Diagnostic Value of NORAD in RPL and UIF

Results of ROC curves showed that the endometrial expression of NORAD could be used to differentiate RPL and UIF with an AUC of 0.977 (95% CI: 0.956–0.999) and 0.970 (95% CI: 0.941–0.998), sensitivity of 0.873 and 0.955, and specificity of 0.845 and 0.948 (Figure 2), respectively.

## 4. Discussion

Placenta is the active interface between mother and fetus, which is related to the rapid development and exposure of molecular markers in the uterus. Genomic imprinting is involved in the development of placenta. For instance, increased mRNA expression of IGF2 and decreased expression of H19 were detected in endometrial tissues of females with UIF [14]. A variety of factors such as chromosomal abnormalities, maternal immunological rejection, and hormonal imbalance are associated with RPL. Normal cellular regulation of these factors is essential for maintaining normal pregnancy, and differential gene expression affects the biological processes of RPL [15]. lncRNAs have attracted extensive attention in disease development because of their enormous diversity in evolutionary conservation, expression level, molecular function, and cellular localization [16]. Previous studies have indicated that lncRNAs including lnc32058, lnc09522, and lnc98497 were differentially expressed in male infertility. Regulation role of lncRNAs on gene expression has been identified in female reproductive disorders [17]. The patients with polycystic ovary syndrome showed elevated expression of lnc-MAP3K13-7:1 in inhibited granulosa cell [18]. HZ07 lncRNA was upregulated induced by benzo(a)pyrene in RPL and overexpression of HZ07 inhibited trophoblast cell migration [19].

Human LINC00657 RNA or alternatively named as NORAD is abundantly expressed in human tissues and cell lines after DNA damage. NORAD was reported as an oncogene of most cancer-related diseases. The role of NORAD in increasing cell viability, proliferation, migration, and invasion while inhibiting apoptosis has been explored in colorectal cancer study presented by Wang et al. [20] and Zhang et al. [21]. Besides, Yang et al. revealed that overexpression of NORAD enhanced migration and invasion of hepatocellular carcinoma cells by suppressing miR-202-5p [22]. However, upregulation of NORAD contributed to suppress tumor growth and enhance apoptosis of endometrial cancer cells. The effects have been exerted through interaction between NORAD and far upstream element binding protein 1 (FUBP1), resulting in attenuation of nuclear localization of this anti-apoptotic protein and releasing pro-apoptotic gene promoters [23]. In this study, we compared the relative expression of NORAD in endometrial tissues from females with UIF, females with RPL, and fertile females. The qRT-PCR manifested that lower expression of NORAD was detected from females with UIF and females with RPL compared with females with normal fertility. UIF and RPL females showed no significant difference concerning NORAD expression. Abnormal female hormone levels lead to negative impact on the reproductive system. FSH is the most commonly used indicator in determining ovarian reserve and represents an indispensable part of fertility treatment [24]. LH plays a vital role in role in promoting follicular growth and maturation in ovarian function. It can be used as an effective predictor of ovarian function when it is combined with FSH [25]. P is essential for the establishment and maintenance of pregnancy through its role in endocrine and immunity [26]. This study found that the fertile females had lower level of FSH, LH, T, PRL, and E2 in serum but showed higher P level than the females with either UIF or RPL. A slight difference in these hormones was noted in females with UIF and females with RPL. Furthermore, Pearson correlation analysis in our study also confirmed that no correlations were identified between NORAD expression and these hormones levels except for E2, whereas E2 level was negatively correlated with NORAD expression. Lastly, we detected the diagnostic value of NORAD in RPL and UIF and found that NORAD yielded AUC of 0.977 and 0.970, respectively, for differentiating RPL and UIF.

However, some limitations should be noted in this study. First, the study consisted of bioinformatics analysis, and qPCR experiment, RNA-sequencing, or arraying in included endometrial tissues will be required in further study. Second, small sample size used for NORAD expression relation to RPL and UIF may reduce reliability of results. Third, there is no evidence presenting the discriminatory nature of this lncRNA in RPL or UIF, and the functions of this lncRNA are yet unclear. Finally, two different datasets were used in the study, but how their endometrial tissues were collected remains unclear.

In conclusion, the present study identified that NORAD expression in endometrial tissues was associated with the occurrence of UIF and RPL in females, and negative correlation was observed between E2 level in serum and NORAD expression. The result may trigger a series of special diagnostics and treatment options for females with UIF and RPL.

## Figures and Tables

**Figure 1:** Low endometrial expression of NORAD in RPL and UIF. (a) The relative expression level of NORAD in the endometrial tissues obtained from women with UIF (*n* = 32), women with RPL (*n* = 48), and fertile women (*n* = 62) was quantified by qRT-PCR. (b) Pearson correlation analysis of the serum level of E2 and the relative expression level of NORAD in the endometrial tissues of UIF. (c) Pearson correlation analysis of the serum level of E2 and the relative expression level of NORAD in the endometrial tissues of RPL.

**Figure 2:** ROC curves of the endometrial expression of NORAD used to differentiate RPL and UIF.

**Table 1:** Identification of differentially expressed RNAs in the endometrial samples between women with RPL and fertile women and between women with UIF and fertile women.

Gene symbol	GB_ACC	Log2FC	RPL or UIF vs. control
NORAD	NR_027451	−1.53	RPL vs. control
ZNF90	AK298173	−1.24	RPL vs. control
SUMO1P3	NR_002190	−1.14	RPL vs. control
ANXA2	NM_001002857	−1.12	RPL vs. control
CAPZA2	NM_006136	−1.05	RPL vs. control
SFRP4	NM_003014	−1.21	RPL vs. control
NORAD	NR_027451	−1.20	UIF vs. control
MAGEA6	NM_175868	−1.06	UIF vs. control
RNA18SN5	NR_003286	1.08	UIF vs. control

NORAD, non-coding RNA activated by DNA damage; ZNF90, zinc finger protein 90; SUMO1P3, SUMO1 pseudogene 3; ANXA2, annexin A2; CAPZA2, capping actin protein of muscle Z-line subunit alpha 2; SFRP4, secreted frizzled related protein 4; MAGEA6, MAGE family member A6; RNA18SN5, RNA, 18S ribosomal N5.

**Table 2:** Demographics and clinical characteristics of women with UIF, women with RPL, and fertile women.

Characteristics	UIF (*n* = 32)	RPL (*n* = 48)	Normal fertility (*n* = 62)
Age (year)	30.56 ± 4.83	29.06 ± 4.17	29.45 ± 4.45
BMI	23.72 ± 3.03	23.51 ± 3.11	22.68 ± 2.87
History of taking oral contraceptives (*n*(%))	10 (31.25%)	18 (37.50%)	15 (24.19%)
History of algomenorrhea (*n*(%))	15 (46.88%)	22 (45.83%)	23 (37.10%)
History of family history (*n*(%))	2 (6.25%)	2 (4.15%)	2 (3.22%)
FSH (mIU/ml)	6.29 ± 2.07^*∗*^	6.62 ± 2.11^*∗*^	4.40 ± 1.30
LH (mIU/ml)	7.79 ± 2.33^*∗*^	8.37 ± 2.50^*∗*^	5.80 ± 2.05
T (nmol/L)	1.74 ± 0.30^*∗*^	1.80 ± 0.32^*∗*^	1.45 ± 0.28
PRL (mIU/L)	493.81 ± 150.03^*∗*^	501.73 ± 149.69^*∗*^	316.47 ± 120.03
E2 (pmol/L)	115.47 ± 38.12^*∗*^	120.72 ± 41.55^*∗*^	81.63 ± 29.04
P (nmol/L)	1.05 ± 0.41^*∗*^	0.95 ± 0.30^*∗*^	2.53 ± 0.80

BMI, body mass index; FSH, follicle stimulating hormone; E2, estradiol; P, progesterone; LH, luteinizing hormone; T, testosterone; PRL, prolactin; ^*∗*^*P* < 0.001 compared to normal fertility, analyzed by independent Student's *t*-test.

## Data Availability

The dataset (accession number: GSE165004) analyzed during the current study is available in the Gene Expression Omnibus (https://www.ncbi.nlm.nih.gov/geo/query/acc.cgi?acc=GSE165004). Other data used to support the findings of this study are included within the article.
